# Research on Characteristic of Chronic Spontaneous Urticaria Based on Multiscale Entropy

**DOI:** 10.1155/2021/6691356

**Published:** 2021-05-25

**Authors:** Shujuan Wang, Ping Song, Rong Ma, Yanzhong Wang, Bin Yu, Min Wang, Meiqi Wang, Jihong Shen, Yuntao Dai, Yuming Wang, Wanqing Xie

**Affiliations:** ^1^College of Mathematical Sciences, Harbin Engineering University, Harbin 150001, China; ^2^Department of Dermatology, Guang'anmen Hospital, China Academy of Chinese Medical Sciences, Beijing 100053, China; ^3^School of Population Health & Environmental Sciences, Faculty of Life Science and Medicine, King's College London, London, UK; ^4^Suzhou Fanhan Information Technology Co., Ltd, China

## Abstract

Chronic spontaneous urticaria (CSU) is a common skin disease which symptom is local pruritus and pain. In medicine, researchers take a certain point that the brain is the control center of CSU, but in previous experiments, the researchers found that cerebellum also had a certain effect on CSU. In order to find out the influence of CSU in the brain and cerebellum, we collected the brain resting-state fMRI data from 40 healthy controls and 32 CSU patients and used DPABI to preprocess. We calculated the entropy values of five scales by using multiscale entropy (MSE) and the average entropy values of two groups' BOLD signals; 15 regions with significant differences were found which not only had a more detailed impact in the brain but also had an impact in the cerebellum, such as precentral gyrus, lenticular putamen, and vermis of cerebellum. In addition, we found that compared with the healthy controls, the entropy values of CSU patients showed two trends which need further study. The advantage of our experiment is that the multiscale entropy value is used to get more influence regions of CSU in the brain and cerebellum. The results of this paper may provide some help for the pathological study of CSU.

## 1. Introduction

Chronic spontaneous urticaria (CSU) is a disease, characterized by recurrent (<24 h) pruritic wheal of skin and mucous membranes, with a duration of more than 6 weeks, and spontaneous, temporary, and itchy recurrent episodes that occur several times a day to several days [1]. Studies have shown that CSU can have a significant impact on the lives of patients, including daily work and mental health [2, 3]. According to the statistical population, the prevalence of CSU is about 0.5%-1% [4]. In view of the similar allergic reactions in patients with chronic spontaneous urticaria, in most cases, the triggering factor cannot be determined. There are several theories of pathogenesis, but there is no reliable theoretical proof [5]. Because the pathogenesis of CSU is not clear, the current treatment options are limited [6]. Before 2014, antihistamines were the only approved drugs by CSU, and 50% of patients still have symptoms after treatment [4].

The clinical manifestations of CSU are pruritus [7], which sends signals to the brain through the spinal cord [8], and the brain is the control center for pruritus. The pathogenesis of CSU is complex and unclear. From a systemic perspective, complexity reflects the brain's ability to adapt to environmental change, which can be compromised in CSU, leading to abnormal skin itching, which may patients with impaired mental function [9]. Therefore, studying the complexity of brain activity may provide advice on how CSU correlates with the pathophysiology of brain function. According to the study, the BOLD signals measured by resting-state functional magnetic resonance imaging (rs-fMRI) is the hemodynamic response of a large number of nerve cells [10], which is the best tool for us to understand the brain. In recent decades, studies have analyzed the functional connectivity data of different brain regions to obtain local connectivity of brain regions and spontaneous local brain activity characteristics [11], such as seed-based resting state functional connectivity [9] and Regional homogeneity (ReHo) [12]. ReHo can be used to describe the local consistency of time series of adjacent voxels in a region. Studies have used such methods to explore different ways of connecting different brain regions or networks to help locate brain regions associated with related diseases [13–15]. Wang et al. used ReHo to explore the brain regions associated with itching [16]. Yang et al. understand the brain function of patients by comparing the characteristics and differences of low-frequency amplitude (ALFF) [17] in the brain region at rest status. However, the current link between CSU and the complexity of brain activity remains unrecognized.

Multiscale entropy (MSE) [18] is a method for data with nonstationary and nonlinear features and is widely used in sample complexity calculations. MSE provides the characteristics of entropy across multiple time scales, so that the complexity of the physiological signals not included in the traditional method can be extracted to assess the complexity of the time series of the diseased and healthy groups [19]. MSE has the following advantages: (1) The required length of data is shorter, and the amount of calculation is smaller. (2) The ability to resist noise and anti-interference is better. (3) At a multiscale, a new sequence is constructed based on a given physiological signal sequence, and the analysis is more systematic. Based on the above advantages, multiscale entropy has been used more and more in the field of biomedical signal processing [19]. Many studies have been using MSE to quantify the complexity and regularity of BOLD signals [20–22], such as using the MSE method to analyze the complexity of electroencephalogram (EGG) in patients with Alzheimer's disease and inferring the possibility of MSE from the findings. It is a useful tool for checking the complexity of EEG [19]. Azami et al. found that MSE analysis of EEG signals helped distinguish patients with Alzheimer's disease and healthy individuals and demonstrated the ability of MSE to characterize brain signal complexity in different bands of Alzheimer's disease [21]. Literature 22 points out that under the same conditions, the AUC value of MSE (AUC = 0.76) is higher than that of HRVI (AUC = 0.70) [22]. Jun and Qian-Li first studied the multiscale entropy of the ST segment of ECG. Studies have shown that average MSE values and fluctuations in range of variation may be more effective in revealing heart health [23].

Numerous studies have shown that MSE plays a very significant role in studying the relationship between physiological signals and brain function [20, 22, 23]. In this study, we used MSE to explore the correlation of brain activity between CSU and HCs. We hypothesized that CSU is associated with reduced complexity of multiple time scales. In addition, we study the entropy distribution of BOLD signals in CSU patients and explore the relationship between resting-state brain activity complexity and associated CSU pathology.

## 2. Materials and Methods

### 2.1. Data Collection and Preprocessing

The research protocol has been approved by the Ethics Committee of Guang'anmen Hospital of China Academy of Chinese Medical Sciences. Experiment agrees with the approved guidelines. All subjects signed written informed consent before the study began. The study participants consisted of 72 Han Chinese participants who were recruited from the dermatology clinic at Guang'anmen Hospital in Beijing. There are 40 healthy subjects (8 males and 32 females, age 25-63), and the affected group consisted of 32 patients with chronic urticaria (6 males and 26 females, age 25-65), characterized by a temporary, itchy, unclear itching of 6 weeks or longer. All patients discontinued antihistamine drugs (such as loratadine, desloratadine, fexofenadine, and cetirizine dihydrochloride) and interventions 3 days prior to the scan. During the scan, the patient did not have any itching [24], UAS > 14, and age and gender match. Demographic and clinical data for participants are as shown in Table 1.

### 2.2. Description of Machine Parameters in Functional Magnetic Resonance Scanning

During the experiment, the fMRI scan was performed on a 3.0T Siemens MAGNETOM Skyra MRI system equipped with a 20-channel head coil. All functional magnetic resonance imaging experiments were performed in the morning. Foam pads were used to limit head movement. T2 weighted images to rule out lesions and abnormalities. A high-resolution T1 weighted structure image is obtained by using a three-dimensional fast gradient echo sequence with a repetition time (TR = 5000 ms), an echo time (TE = 2.98 ms), a field of view (FOV = 256 × 240 mm^2^), and a flip angle (FA = 4°). The matrix size is 256 × 256; the slice thickness is 1 mm; the gap is 0 mm, a total of 176 pieces. Using a 43-layer gradient echo plane imaging EPI sequence (TR = 2500 ms, TE = 30 ms, matrix 70 × 70, FOV 210 × 210 mm^2^, FA = 90°), slice thickness 3 mm, gap 0 mm, and collection covering the entire brain, the fMRI image is sliced parallel to the AC-PC line. The scan time was 369 seconds (the first 9 seconds of the virtual scan), and the subjects were asked to close their eyes [24].

### 2.3. Data Preprocessing

The stationary state fMRI image was preprocessed using the data processing assistant DPABI for the stationary state fMRI toolbox implemented in MATLAB (MathWorks, Natick, MA, USA). Preprocessing includes as follows:

1. *Slice Timing*. In the process of fMRI acquisition, since it takes several seconds to collect a whole brain image (i.e., TR = 2.5 s), the image level of the brain is not collected at the same time. In this experiment, there are 43 layers of images in the whole brain. Therefore, the time required to collect one layer is about 0.058 s, and the collection method is compartmental collection, that is, first collect 1, 3, 5, 7,…, 43 layers, and then collect 2, 4, 6,…, 42 layers, so the acquisition between different layers will produce a time difference. The principle of time layer correction is to normalize all layers of the whole brain to the same layer through data processing (usually in the middle layer, layer 43rd); after this processing, the data is easier to study later
2. *Realign*. The purpose of MRI is to scan and image the structural images in the brain, so the subject's subtle head movements will have a great impact on the scan results, and it is impossible to keep the head completely motionless. In this data collection, the head movement tolerance of the subject is less than 2 mm, and the rotation is less than 2 degrees. If the subject is more than 2 mm or rotated more than three millimeters in any direction in a three-dimensional space, it is not allowed
3. *Standardize into the Standard Stereotactic Space of the Montreal Institute of Neurology (MNI) EPI Template and Then Resample to*3 × 3 × 3 *mm^3^ Voxels*. Because of the high and low body weight of other subjects or other reasons, each person's brain size is different, but the human brain structure and its structural positional relationship are unified, so all subjects can be transformed. Get unified. Realigning and normalizing to the MNI space facilitates the study of brain structures and increases the universality of experimental results
4. *Smooth*. Although the purpose of the previous step is to eliminate the effects of different brains, there will be a slight deficiency. The subtle errors are not guaranteed to be completely eliminated. Therefore, after standardization, we will perform another smoothing process. The main purpose is to make each voxel and its surrounding voxels smoother
5. *Filter*. Using bandpass time filtering (0.01–0.08 Hz) to minimize noise. This step can attenuate the noise frequency and improve the signal-to-noise ratio

Due to the instability of the initial fMRI scan, the first 10 data points of each BOLD signals are discarded; therefore, the remaining 134 data points per time series are used for analysis.

### 2.4. Multiscale Entropy Algorithm

#### 2.4.1. Sample Entropy Algorithm

Sample entropy is a kind of entropy commonly used by researchers in the field of physiological signals research in recent years. The advantages are (1) sample entropy can be well applied to shorter time series. (2) The sample entropy is robust to noise. (3) For random time series, the sample entropy has good consistency [25]. Therefore, in this section, we briefly introduce multiscale entropy based on sample entropy. The principle of sample entropy is to measure the complexity of data by using the self-similarity of time series. The basic algorithm flow is as follows: Let the original time series *x*(1), *x*(2), ⋯, *x*(*N*) have *N* data points.

1. A set of *m*-dimension vectors in sequential order of serial numbers:

(1) $$\begin{array}{c} X\left(i\right)=\left[x\left(i\right),x\left(i+1\right),\cdots ,x\left(i+m-1\right)\right],i=1,2,\cdots ,N-m+1. \end{array}$$

(2) Define the distance between *X*(*i*) and *X*(*j*) as the largest difference between the corresponding elements in the two vectors. The formula is expressed as:

(2) $$\begin{array}{c} \text{dist}\left[X\left(i\right),X\left(j\right)\right]=\max\left[\left|x\left(i+k\right)-x\left(j+k\right)\right|\right],k=0,1,2,\cdots ,m-1,j=1,2,\cdots ,N-m+1,j\neq i. \end{array}$$

Calculate the distance between the vector *X*(*i*) and the rest of the vector *X*(*j*).

(3) Give a threshold *r*, for each *i* calculate the number of dist[*X*(*i*), *X*(*j*)] < *r* as *B*_*i*_, get the ratio of this number to the total number of distances:

(3) $$\begin{array}{c} C_{i}^{m}\left(r\right)=\frac{B_{i}}{\left(N-m\right)}. \end{array}$$

(4) Average for all *C*_*i*_^*m*^(*r*):

(4) $$\begin{array}{c} C^{m}\left(r\right)=\frac{\sum C_{i}^{m}\left(r\right)}{N-m+1}. \end{array}$$

(5) Let *m* = *m* + 1, repeat steps 1 ~ 4, get *C*^*m*+1^(*r*):
(6) The sample entropy sequence is:

(5) $$\begin{array}{c} \text{SampEn}\left(x,m,r\right)=-\ln\frac{C^{m+1}\left(r\right)}{C^{m}\left(r\right)}. \end{array}$$

#### 2.4.2. Multiscale Entropy Algorithm

Due to the nonlinearity of the BOLD signals, the single-scale entropy cannot fully measure its complexity. Therefore, we need to measure its complexity on multiple scales [26, 27], and multiscale can be understood as magnifying glass magnification. Multiple different scales will see different characteristics of the signals. The basic entropy algorithm of multiscale entropy uses sample entropy. Experiments have shown that the sample entropy is more suitable for short-time time series, that is, the signal length does not affect the entropy result [25]. The multiscale entropy algorithm consists of two steps: (1) coarse granulation process, that is, multiscale transformation of the original time series; (2) substituting the coarsely granulated new time series into the sample entropy calculation. In order to obtain a coarse-grained time series with a scale factor of 1, first, the original sequence is divided into *τ* nonuniform time windows, and the *k*-th coarse-grained time series is defined as follows:

(6) $$\begin{array}{c} y_{k}^{\left(\tau \right)}=\frac{1}{\tau }\sum x\left(i\right),1\leq k\leq \frac{N}{\tau },i=\left(k-1\right)\tau +1,\cdots ,k\tau . \end{array}$$

When the scale factor is 1, the multiscale entropy after the coarse-grained sequence is the original sample entropy:

(7) $$\begin{array}{c} \text{MSE}\left(x,\tau ,m,r\right)=\text{SampEn}\left(y_{1}^{\left(\tau \right)},m,r\right). \end{array}$$

When the scale factor is *τ*, the length of the sequence after coarse granulation is *N*/*τ* of the original time series.

We can summarize the basic algorithm flow of multiscale entropy: (a) construct a coarse-grained time series according to different scale factors, (b) quantify the sample entropy of each coarse-grained time series, and (c) check the sample entropy within a certain range distribution and statistical results.

We generally require the length of the time series to be 10^*m*^ ~ 30^*m*^. In this experiment, since the original time series is short, we choose the parameter values as *m* = 1, *r* = 0.35*SD*, *τ* = 5 of the MSE [28, 29]. We use the AAL template in the DPABI toolkit to divide the brain into 116 brain regions for complexity analysis. In addition, we standardize the BOLD signals to avoid noise and outlier interference before performing MSE analysis. For the generated entropy values, we combined the statistical method, the general linear model to more scientifically compare the differences between the CSU patients and the healthy controls.

## 3. Results

### 3.1. Clinical Outcome

Analysis of personal information on 32 CSU patients and 40 healthy controls showed no physiological correlation. The patient did not undergo therapeutic intervention, and UAS7 remained at a level of 30.8 ± 6.2.

#### 3.1.1. Comparative Results Display Analysis Based on ALFF (Amplitude of Low Frequency Fluctuation)

The comparison results are generated using the ALFF values of the brain. We use the Student's *t*-test to statistically analyze the ALFF values of healthy controls and CSU patients and then use the Brain View of DPABI to display it.  Figure 1 shows the comparison of the outer side of the cerebral hemisphere, and it can be seen that compared with healthy people, the patient's ALFF values has changed in this place. The following figure shows the comparison of the inner and lateral sides of the cerebral hemisphere. It is obvious that the patient has a significant increase in ALFF values at the position of the lenticular putamen. In order to confirm that all the changed brain regions are related to urticaria, we conducted further multiscale entropy experiments.

### 3.2. Multiscale Entropy Analysis Results Based on BOLD Signals

In order to further explore the parts of the brain that show differences in the above analysis and find out which areas are associated with pruritus by extracting BOLD signals from the healthy controls and the CSU patients. Time series refer to physiological signals displayed by each brain region at each acquisition time. The multiscale entropy analysis is performed on the BOLD signals, and then, the following two different statistical analysis comparisons are performed on the multiscale entropy results.

#### 3.2.1. Multiscale Entropy Analysis Results Using General Linear Models (GLM)

Multiscale entropy was used to perform a GLM test. In the brain, the R precentral gyrus, L superior frontal gyrus, R orbital superior frontal gyrus, L middle frontal gyrus, R middle frontal gyrus, R orbital middle frontal gyrus, R supplementary motor area, L postcentral gyrus, L angular gyrus, L paracentral lobule gyrus, R lenticular putamen, and L superior temporal gyrus have *p* < 0.05, so they have statistical significance. In the cerebellum, the L superior cerebellum, the R superior cerebellum, and the vermis of cerebellum have *p* < 0.05, so they have statistical significance (Table 2).

#### 3.2.2. Analysis Results with Different Scale Comparison

The multiscale entropy of the same brain region in the healthy controls and CSU patients was analyzed and found. There were two trends in the change of the entropy values between the CSU patients and the healthy controls: (1) The entropy of healthy controls at five scales is always higher than that of CSU patients; (2) The entropy value of CSU patients at five scales is higher than that of the healthy controls at the same scale (Figure 2).

## 4. Discussion

In this study, we investigated changes in ALFF values in patients with chronic urticaria compared to healthy controls. We obtained the consistent conclusion as Yuming Wang [16] by using the Student's *t*-test: the patient showed a significant increase in ALFF values in the lenticular putamen. Similarly, it is difficult to get other more detailed significant areas. To get more accurate results, the multiscale entropy is chosen to measure the complexity of the nonlinear BOLD signals.

The clinical manifestations of CSU are pruritus or tingling of the skin. Itching is a physiologically pleasing behavior that is related to the intensity of itching [30, 31]. This pleasant experience is controlled by an active brain area and will show a sense of pleasure even without scratching. In previous studies [16], these areas were considered to be activated: the R precentral gyrus, L superior frontal gyrus, R supplementary motor area, L postcentral gyrus, L angular gyrus, R orbital superior frontal gyrus, R orbital middle frontal gyrus, lenticular putamen, and the L superior temporal gyrus. The precentral gyrus is the location of the primary motor cortex, which is the main area of the motor system and works in conjunction with other brain regions to plan and perform scratching movements. Studies show that primary somatosensory cortex is related to itching [16]. The postcentral gyrus is the somatosensory area of the human body. Studies have shown that the primary somatosensory area is related to pruritus management [16]. According to previous studies, with functions of memory, judgment, analysis, thinking, and operation of the prefrontal lobe [32], R lenticular putamen [33] and L superior temporal gyrus [34] are related to itching. According to research, the sensitivity of peripheral and central neurons to pain and pruritus has shown striking similarities [35]. The angular gyrus is a visual language center, which is related to the cognitive function network and affects the pain matrix [33]. Therefore, we speculate that the angular gyrus is related to itching.

In this study, we found that CSU is associated with the L middle frontal gyrus and R middle frontal gyrus, showing a reduction in complexity. The middle frontal gyrus is one of the components of prefrontal lobe and plays a vital role in cognitive function. Previous research has also shown that the middle frontal gyrus may involve psychological responses such as sensory-resolved processing, emotional response, motor planning, and cognitive evaluation [32]. Thereby achieving advanced central treatment of pruritus. CSU may be related to the reduced complexity of the paracentral lobule gyrus [36]and the activity of the brain regions of the vermis of cerebellum [33]. The central lobular lobe belongs to the first somatic motor area and is closely related to the action of pruritus and scraping. Studies have shown that the vermis of cerebellum are associated with pain [33], while many interactions between itching and pain in the process of transmission and sensitization, the pain caused by scratching will reduce itching, and vice versa [37]. From this, we suspect that the vermis of cerebellum are related to itching. We also found that the complexity of the L superior cerebellum and R superior cerebellum was increased in patients. The cerebellum is an important regulatory center of movement, and there are a large number of afferent and efferent connections. Neuroanatomical studies showed that the cerebellum sends projections to the cortical sensory motor area and reward region via the thalamus, which indicates that the cerebellum may participate in the neuropathological process of CSU [16].

In addition, we investigated the differences in the complexity of brain activity between CSU patients and healthy controls for brain areas with significant entropy values. We plotted MSE curves on five scales and found the following two cases: one is that the entropy value of the healthy controls is greater than the entropy values of the CSU patients on each scale, such as R precentral gyrus, L superior frontal gyrus, R middle frontal gyrus, R middle frontal gyrus orbital part, R supplementary motor area, L postcentral gyrus, L angular gyrus, paracentral lobule, and vermis of cerebellum. We can conclude that in the above brain regions, the complexity of the BOLD signals in the healthy controls is higher than the complexity of the BOLD signals in the CSU patients. Another case showed that the MSE values of the CSU patients in superior frontal orbital part, lenticular nucleus putamen, superior temporal gyrus, and superior cerebellum were higher than that of the healthy controls on all scales. The orbital frontal gyrus participates in the prefrontal cortex's integration function, which is related to advanced activities such as thinking. And some studies have shown that the prefrontal lobe plays a major role in the perception and expectation of pain [38]. The lenticular nucleus, as part of the striatum, is related to the emotional processing of painful stimulation and is also a brain region related to reward [39]. The superior temporal gyrus is related to memory function, but there is also relevant literature indicating that the temporal lobe can be deactivated when it is stimulated by related pain [34]. These three brain regions may be involved in the perceptual processing of painful stimuli caused by itching, which in turn can activate them. These findings may provide valuable insights into the neuropathology of chronic urticaria.

## 5. Conclusion

Using multiscale entropy analysis, we assessed the abnormalities of resting brain activity in patients with pruritus and their pathological relationship with disease. Our findings represent a new perspective on functional brain activity in pruritus. At the same time, we have also found that parts of the cerebellum also have an effect on pruritus, which enhances the understanding of various pathophysiological processes in pruritus. Further, the use of entropy analysis in the time dimension can facilitate clinical disease imaging markers.

## Figures and Tables

**Figure 1:** The change in the level of ALFF indicates that urticaria appears in the brain as activation of part of the brain and inhibition of part of the brain.

**Figure 2:** A graph of two trends. The (a) expresses the right orbital superior frontal gyrus which belongs to case 2; complexity of BOLD signals in this area is higher than that in healthy person; this situation also existences in lenticular putamen, superior temporal gyrus, and the two areas of the superior cerebellum. The (b) expresses the right R orbital middle frontal gyrus which belong to case 1; the complexity of BOLD signals in this area is lower than that in healthy person; this is consistent with human characteristics; other sick areas belong to this situation.

**Table 1:** Demographics and clinical characteristics.

Variables	CSU (*n* = 32)		HC (*n* = 40)	
	Mean	SD	Mean	SD
Age	47.25	11.88	43.35	11.11
Gender, female	26	81.25%	32	80%
Handedness, right		100%		100%
UAS7	30.8	6.2		

Categorical data are given as number (%).

**Table 2:** Regions showing significant changes in the MSE complexity profiles of BOLD signals from patients with CSU.

Brain regions	MNI coordinates			*F* value	*p* value
	*X*	*Y*	*Z*		
R precentral gyrus	40.37	-8.21	52.09	29.895	0.005
L superior frontal gyrus	-19.45	34.81	42.20	19.330	0.012
R orbital superior frontal gyrus	17.49	48.10	-14.02	25.257	0.007
L middle frontal gyrus	-34.43	32.73	35.46	10.804	0.030
R middle frontal gyrus	36.59	33.06	34.04	10.566	0.031
R orbital middle frontal gyrus	32.18	52.59	-10.73	17.302	0.014
R supplementary motor area	7.62	0.17	61.85	13.996	0.020
L postcentral gyrus	-43.46	-22.63	48.91	11.000	0.029
L angular gyrus	-45.14	-60.82	35.59	12.034	0.026
L paracentral lobule gyrus	-8.63	-25.36	70.07	8.299	0.045
R lenticular putamen	26.78	4.91	2.46	8.331	0.045
L superior temporal gyrus	-54.16	-20.68	7.13	38.042	0.004
L superior cerebellum	-10.95	-48.95	-45.90	9.193	0.039
R superior cerebellum	9.46	-49.50	-46.33	11.496	0.028
Vermis of cerebellum	1.15	-64.43	-34.08	8.087	0.047

All brain clusters have *p* < 0.05 corrected for GLM. ^a^L: left; R: right. ^b^(*x*, *y*, *z*) was the coordinate of each brain region. ^c^Volume was computed from cluster size (3∗3∗3 mm^3^ voxel).

## Data Availability

The copyright of the data used in this paper belongs to Guang'anmen Hospital. We signed a written informed consent with the patient before the study and hid the information of all patients in the study. So it cannot be disclosed without authorization.
